# The Way of Severe Nursing of Respiratory System Failure

**DOI:** 10.1155/2021/1667458

**Published:** 2021-10-29

**Authors:** Qiongshan Liu, Weichao Li

**Affiliations:** ^1^The Seventh Affiliated Hospital, Sun Yat-Sen University, Guangzhou, China; ^2^The Office of Organ Donation and Transplant, Sun Yat-Sen University, Guangzhou, China; ^3^Infectious Diseases Department, Sun Yat-Sen University, Guangzhou, China

## Abstract

Respiratory failure is the most common clinical symptom, seriously endangering people's health, which is mainly caused by a series of reasons, leading to serious respiratory dysfunction and severe pulmonary respiratory disorders, damaging the pulmonary airway function, and causing disability to maintain normal human gas exchange activities. At present, the main treatment of respiratory failure is to use the ventilator to help patients exchange gas and keep their breathing unobstructed. The nursing method is also around the artificial airway mechanical ventilation. The nursing of patients with respiratory failure is mainly respiratory nursing and psychological nursing. In this paper, the main research is to explore the way of severe nursing of respiratory failure. Before the nursing of respiratory failure, we should carry out nursing detection of the ventilator and test its performance, tightness, pipeline safety, and airway patency. Then carrying on the respiratory failure mechanical ventilation nursing and clarifying its mechanical ventilation nursing process is the main work of intensive care, at the same time, giving consideration to the psychological nursing of respiratory failure and implementing comprehensive nursing. In this paper, 50 patients were selected and divided into group A and group B; group A was given comprehensive nursing, and group B was given general nursing. The experimental results show that a series of situations in group A are more optimistic than those in group B. There was no doubt that the PH value of the two groups changed significantly 6 months after discharge. The pO_2_ value of group A was higher than that before discharge, while the pCO_2_ value of group B was unstable and increased. The pO_2_ value of group A was 55.52 before discharge and 62.36 six months after discharge. The pCO_2_ value of group A was 54.31 before discharge and 50.61 six months after discharge. The pCO_2_ value of group B was 55.23 before discharge and 57.34 six months after discharge.

## 1. Introduction

Respiratory failure is caused by a series of reasons, leading to serious respiratory dysfunction and severe pulmonary respiratory disorders and causing disability to maintain the normal human respiratory gas exchange activities of clinical symptoms, a serious threat to people's lives [1, 2]. At present, when patients with respiratory failure enter ICU for emergency rescue nursing, the method is to use ventilator and respiratory tube for mechanical ventilation and use machine for artificial oxygen supply [3, 4]. The basic principle of mechanical ventilation in the treatment of respiratory failure is to strengthen respiratory support, including maintaining the smooth airway, eliminating hypoxia, improving respiratory conditions, and strengthening the supervision and support of the whole organ treatment [5, 6]. In the nursing process of patients with respiratory failure, it is mainly to carry out respiratory nursing for patients, test their respiratory state, and then carry out psychological nursing for patients and their families, comforting and encouraging patients to provide emotional support [7, 8]. In this paper, the key to explore the critical care approach of respiratory system failure is mechanical ventilation nursing, through the use of mechanical devices to replace the patient's own assisted breathing, provide oxygen through the ventilator into the breathing pipe, and boost breathing activities [9, 10]. Note that respiratory failure is a serious clinical disorder caused by various reasons of pulmonary ventilation and/or ventilation dysfunction, which leads to ineffective gas exchange and hypoxia with (or without) carbon dioxide retention, resulting in a series of physiological functions and metabolic disorders.

In the research on the approach of severe care of respiratory system failure, many scholars at home and abroad have studied it and achieved certain research results. Some scholars pointed out that the rational use of ventilator, active and effective treatment, and nursing can effectively control the symptoms of patients, increase exercise endurance, reduce the occurrence of complications, reduce the number of hospitalizations, and prolong the life of patients [11]. Other scholars have pointed out that the complications of respiratory failure are closely related to the time of receiving ventilator treatment and the difficulty of weaning, and the consequences are increased mortality, increased costs, and decreased quality of life [12]. The causes of respiratory failure include respiratory diseases, lung tissue diseases, pulmonary vascular diseases, thoracic diseases, and respiratory muscle diseases of nerve center and its conduction system. The causes of thoracic lesions are thoracic trauma, surgical trauma, pneumothorax, and pleural effusion, which affect thoracic activity and lung expansion, leading to ventilation reduction and uneven inhalation of gas affecting ventilation function.

This paper mainly studies the way of severe nursing of respiratory system failure. Before the nursing of respiratory failure, the ventilator was tested for its performance, tightness, pipeline safety, and airway patency. Then this article carries on the respiratory failure mechanical ventilation nursing and clarifies its mechanical ventilation nursing process, which is the main work of intensive care. At the same time, it also gives consideration to the respiratory failure psychological nursing and implements comprehensive nursing. In this paper, 50 patients were selected and divided into group A and group B. Group A was given comprehensive nursing, group B was given general nursing, and then the situation of patients was studied and analyzed to understand the nursing effect. Respiratory failure is mainly acute and chronic according to the course of disease. Acute respiratory failure refers to the sudden clinical manifestations of respiratory failure caused by the sudden causes of the above five causes, such as cerebrovascular accident, drug poisoning, inhibition of respiratory center, respiratory muscle paralysis, and pulmonary infarction, all of which if not rescued in time, the patient's life will be endangered. Chronic respiratory failure is more common in chronic respiratory diseases, such as chronic obstructive pulmonary disease and severe pulmonary tuberculosis.

## 2. Research on the Way of Severe Nursing of Respiratory System Failure

The examination of respiratory failure mainly includes blood gas analysis, electrolyte examination, sputum examination, pulmonary function examination, and chest imaging examination. It is mainly determined by sputum smear and bacterial culture, which is conducive to guiding medication.

### 2.1. Ventilator Care Testing

#### 2.1.1. Performance Test

Mechanical ventilation devices include ventilator and artificial airway catheter, whose performance is directly related to the effect of respiratory support and the life of patients. During the inspection, first connect the air source and power supply, connect the whole set of external pipes, including humidifier and simulated lung, test the machine with electricity, observe the working state of the machine, adjust the parameters according to the needs, run for about 20 minutes, and then check whether the set parameters and display parameters are consistent and stable.

#### 2.1.2. Airtight Test

To test the airtightness of air bag in front of endotracheal intubation or tracheotomy catheter and the airtightness of ventilator connecting pipe is the basic link to ensure the effect of mechanical ventilation. The main function of the air bag is to close the airway and prevent gas leakage during ventilation. The ideal air bag pressure is the minimum pressure for effectively closing the gap between the air bag and the trachea, which is generally maintained in the range of 20–25mmhg. Clinically, it is very necessary to monitor the pressure of the air bag, usually every 4–8 hours.

#### 2.1.3. Pipeline Safety Inspection

For patients with mechanical ventilation, it is important to ensure the correct and proper fixation of the catheter to prevent accidents caused by catheter displacement. For endotracheal intubation, it is necessary to determine the correct position and depth of the catheter, auscultate whether the respiratory sounds on both sides of the lung are normal, and confirm that the catheter is in the general trachea. After that, fix the catheter with adhesive tape in the shape of “X” or “Y” and record the depth of the catheter tip from the incisor teeth. Generally, the depth is 22–23 cm for men and 21–22 cm for women. The position of conduit shall be monitored, recorded, and handed over every shift. Special attention should be paid to the skin pressure at the contact part with the catheter and cloth belt to prevent the formation of pressure ulcer. When the ventilator pipeline is disconnected from the intubation, the catheter end shall be fixed, and the connection shall not be forcibly disconnected to prevent the catheter from shifting. When carrying out various nursing operations, it is necessary to release the constraints under the condition of ensuring the safety of patients, so as to avoid accidental extubation. When changing the patient's position, attention should be paid to adjusting the position of the catheter and the ventilator pipeline, and turning the patient's head, neck, and trunk in a straight line to prevent accidents caused by catheter displacement and prolapse.

The functions of the ventilator mainly include the degree of computerization of the ventilator, screen prompt in case of failure, perfect alarm function, sputum suction function, atomization function, and breath holding function. Among them, perfect alarm functions, such as oxygen supply, gas supply, minute ventilation, upper pressure limit, lower pressure limit, respiratory rate, tidal volume, asphyxia ventilation, background ventilation setting, machine disconnection, air leakage, flow sensor, working state, and oxygen flow, ensure the safety of mechanical ventilation process. The clinician can adjust the alarm range set by the parameters according to the patient's state.

### 2.2. Nursing of Mechanical Ventilation in Patients with Respiratory Failure

1. Select the ventilator in good working condition, set the parameters, select ST mode, and set the positive end inspiratory pressure and positive end expiratory pressure according to the original invasive ventilator parameters.
2. Connect the noninvasive ventilator pipeline correctly, remove the nasal mask or nasal mask at the end of the noninvasive ventilator pipeline, connect the noninvasive ventilator pipeline to the simple respirator check valve, pay attention to the direction of the simple respirator check valve, connect the intubation tube, and connect the noninvasive ventilator with the nasal intubation tube. The one-way valve of the simple respirator has an oxygen suction side hole, which is connected to the central oxygen supply device through an oxygen suction pipe. The setting of oxygen flow is mainly adjusted according to the oxygen saturation of the patient's electrocardiogram monitoring finger.
3. During the period of noninvasive mechanical ventilation with noninvasive ventilator, the degree of cooperation between patients and noninvasive ventilator, sputum condition, changes of finger pulse oxygen saturation, and patients' mood were closely observed to guide patients to cooperate with breathing and keep man-machine synchronization.
4. Regarding extubation of nasotracheal intubation, sequential nasal mask, or nasal mask noninvasive mechanical ventilation, the parameters of noninvasive ventilator before extubation were ST mode, IPAP 8–15cmH_2_O, EPAP 4 ∼8cmH_2_O, FIO_2_ ≤ 40%. The patients adapt to the ventilation mode of noninvasive ventilator, and the man-machine cooperation is good; the results of arterial blood gas analysis showed that PaCO_2_ < 50 mmHg, PaO_2_ > 60 mmHg, and SpO_2_ > 90%. Before extubation, prepare the noninvasive ventilator in good working condition, set the parameters of the ventilator, select ST/S mode, that is, select ST or S mode during the day, and select ST mode when sleeping at night. Pull out the endotracheal intubation and then wear the breathing oxygen mask connected with the aerobic tube to the patient's face. After the patient adapts for a moment, connect the ventilator pipeline, turn on the ventilator, and carry out noninvasive mechanical ventilation. During the whole process, closely observe the patient's condition, including mental state, patient's tolerance after connection mode change, man-machine cooperation, cough, expectoration ability, and finger pulse oxygen saturation, and recheck arterial blood gas analysis.
5. On the premise that patients show tolerance and their vital signs are stable, we should gradually shorten the use time of noninvasive ventilator and use nasal catheter for oxygen inhalation. The general vital signs of the patients were monitored: SpO_2_ ≥ 90%, heart rate <100 beats/min, and breathing <35 beats/min. There was no significant change in blood gas analysis. Finally, noninvasive mechanical ventilation was stopped and a nasal catheter was used for oxygen inhalation.

In addition, adjustment of modern ventilators changes the past multiknob single function and adopts the adjustment mode of single knob, which is convenient for clinical use. Digital adjustment is adopted to increase the accuracy of parameter setting. At the same time, clinicians are required to have rich theoretical and practical experience in order to make the parameter setting more in line with the patient's condition. The ventilator also stipulates the safety range of conventional parameters, which needs to be confirmed beyond the range, increasing the safety of mechanical ventilation. Due to the enhanced monitoring and display function of ventilator, the set parameters are clearly displayed, which is conducive to clinicians to evaluate the condition of patients, and can be transmitted through the network. It is also convenient to manage and guide the treatment of mechanical ventilation.

### 2.3. Psychological Nursing of Respiratory Failure

#### 2.3.1. Health Education

The survey found that most patients with respiratory failure will have a relaxed psychology after surgery, which will reduce their compliance of postoperative treatment. Therefore, after the operation of patients with respiratory failure, the nursing staff should timely carry out health education; explain the significance, method, and effect of respiratory failure nursing after the operation; and at the same time, focus on introducing the cases of treatment failure due to lack of cooperation with nursing after the operation, so that they can realize the importance of respiratory failure treatment after the operation, to improve the treatment compliance.

#### 2.3.2. Psychological Counseling

During the period of intensive care, the nursing of patients with respiratory failure needs to plug in the ventilation pipe for respiratory assistance. The medical staff should communicate with the patients and their families more to ease the patients' emotions and give encouragement and support to the patients' families in the daily nursing dialogue to help the patients adjust their emotions. They also should do a good job in working with patients and their families and encourage patients to improve their confidence in treatment and rehabilitation.

#### 2.3.3. Discharge Guidance

Before the patients with respiratory failure go home for home oxygen therapy, the nursing staff should carry out health education and training on the use of ventilator for the patients and their families, set the pressure of noninvasive ventilator, and carry out adaptive treatment in hospital for 3–5 days. The patients will continue to use it at home after discharge and follow up regularly. The patients in the control group were provided with medical oxygen storage tank and flow meter for home oxygen therapy. The patients and their families were taught how to switch on and off the ventilator and the primary adjustment steps; how to wear the mask correctly; and how to disinfect and maintain the ventilator, pipeline, and mask.

At the same time, the application of appropriate amount of stimulants such as doxorubicin can reduce airway edema and control airway edema. However, while respiratory stimulants increase ventilation, they also increase respiratory work and increase metabolic rate, so the effect of increased ventilation may be offset. Long-term application causes respiratory muscle fatigue, and the gain is not worth the loss.

### 2.4. Mean ± Standard Deviation Algorithm for Data Analysis

Efficiency evaluation refers to a series of qualitative and quantitative efficiency evaluation indexes to comprehensively evaluate the clinical practice effect of patients in the standby stage and operation stage and results of mechanical ventilation, so as to analyze and judge the energy efficiency of ventilator and artificial airway under the action of nurses. Through efficiency evaluation, it is conducive to make effective identification of key indexes of mechanical ventilation efficiency, promoting the quality of critical care practice. In this paper, the data of respiratory failure treatment and nursing were analyzed by Excel. The comparison between groups was performed by *t*-test, and the measurement data were expressed by mean ± standard deviation (*x* ± *s*). If *P* < 0.01, the difference was statistically significant; if *P* > 0.05, the difference was not statistically significant; and if *P* < 0.05, the difference was statistically significant.

Standard deviation is most commonly used in probability statistics as a measure of statistical dispersion. The definition of standard deviation is the square root of the arithmetic mean of the square of the deviation between the standard value of each unit and its mean. It reflects the degree of dispersion between individuals in the group. The results measured to the degree of distribution have two properties in principle. It is a nonnegative value with the same unit as the measurement data. There is a difference between the standard deviation of a total amount or the standard deviation of a random variable and the standard deviation of the number of samples in a subset.

Mean is mainly used to find the average of all data in a group of data. In this paper, it is used to study and calculate the treatment of patients with respiratory failure. N is the number of samples of patients with respiratory failure. The specific algorithm formula is as follows:

(1) $$\begin{array}{c} \bar{X}=\frac{\sum {}_{i=1}^{n}X_{i}}{n}. \end{array}$$

Standard deviation, as the arithmetic square root of the arithmetic mean of the square of the mean deviation, is often used as the measurement basis for the statistical distribution degree. In this paper, the direction of treatment degree of patients with respiratory failure is studied. The specific algorithm formula is as follows:

(2) $$\begin{array}{c} \sigma =\sqrt{\frac{\sum {}_{i=1}^{n}{\left(x_{i}-\bar{x}\right)}^{2}}{n}}. \end{array}$$

## 3. Research and Analysis

### 3.1. Research Objects

The research objects of this paper are 50 patients with respiratory failure caused by primary diseases who are hospitalized for intensive care, and the situation is shown in Table 1. Among the patients with respiratory failure, there were 30 male patients and 20 female patients who were undergoing comprehensive treatment and nursing, such as mechanical ventilation, anti-infection, and nutritional support. The patients were stable and had spontaneous breathing, but it was difficult to get off-line, so they still needed certain conditions of respiratory support. In addition, questionnaire method is widely used in social survey at home and abroad. Questionnaire refers to the form used for statistics and investigation to express questions in the form of questions. Questionnaire method is a method that researchers use to do controlled measurement of the research problems, so as to collect reliable data. Questionnaires are mostly sent by mail, individual distribution, or collective distribution. The respondents fill in the answers according to the questions in the form. Generally speaking, the questionnaire is more detailed, complete, and easy to control than the interview form. The main advantages of the questionnaire method are standardization and low cost. Because the questionnaire method is based on the designed questionnaire tools, the design of the questionnaire is required to be standardized and measurable. The 50 patients were randomly divided into group A and group B, 25 people in each group. Group A was given comprehensive nursing care, respiratory nursing, and psychological nursing during treatment, while group B was given routine nursing. The safety and feasibility of the study were explained for the patients and their families. All patients followed the principle of voluntary clinical trials.

### 3.2. Research Process Steps

S/*T* (PSV/PCV + PEEP) mode was used in all patients. The initial EPAP was 2-4cmH_2_O, and IPAP was 8–12cmH_2_O (RR10-16bpm). The pressure was adjusted according to the above monitoring indexes; 2-4cmH_2_O was added every time, evaluated, and adjusted every 6 minutes, and IPAP-EPAP > 4cmH_2_O was maintained.

Monitoring of vital signs during the test included changes of consciousness and mental state, fluctuation of average blood pressure ≥20 mmHg, acceleration of heart rate >20, and respiratory rate >30 or <10 beats/min. Monitoring of respiratory state included respiratory rate >30 or <10 times/min, obvious enhancement of chest breathing or contradictory movement of chest and abdomen, and enhancement of auxiliary respiratory muscle activity. Finger pulse oxygen saturation monitoring: SpO_2_ < 85%. In case of the above situation, the ventilator parameters should be adjusted or suspended immediately.

At the same time, attention should be paid to avoid air leakage: select the mask with appropriate size, adjust the mask and fix the belt to the best position, and ensure that the air leakage is less than 40L/min. The tightness of the headband is appropriate, the use time is more than 6h per day, try to ensure continuous wearing at night, select the appropriate minimum pressure level, encourage expectoration, and give manual assistance when necessary. During the family treatment, keep in touch with the guidance physician to ensure timely and correct adjustment of parameters. The patients in the control group were given propaganda and education before discharge. They were required to use compressed oxygen to connect nasal catheter or nasal obstruction for home oxygen therapy after discharge. The concentration of inhaled oxygen was less than or equal to 30%. They were applied for more than 12 hours a day, humidification was strengthened, continuous oxygen therapy was ensured at night, and they were returned to the hospital for reexamination on the specified date.

## 4. Experimental Study and Analysis on the Way of Severe Nursing for Respiratory System Failure

### 4.1. Analysis of Gender Influence in Patients with Respiratory Failure

For patients with respiratory failure, the main treatment is mechanical ventilation, and respiratory nursing is also a major focus in nursing. The total score of mechanical ventilation system efficiency evaluation is taken as the dependent variable, and the influence of gender on patients with respiratory failure is analyzed to study whether it has statistical significance. The data of patients with respiratory failure who participated in this study were compared, and the results are shown in Table 2. In physics, for multifactor (multivariable) problems, the method of controlling factors (variables) is often used to turn multifactor problems into multiple single factor problems. Each time, only one factor is changed, while the other factors are controlled to remain unchanged, so as to study the impact of the changed factor on things, study them separately, and finally solve them comprehensively. This method is called the control variable method. It is an important thinking method in scientific exploration, which is widely used in various scientific exploration and scientific experimental research.

It can be seen from Table 2 that there is no significant difference in the effectiveness of mechanical ventilation system between patients of different genders (*P* > 0.05), and there is no significant difference in the effectiveness of mechanical ventilation system between patients of different genders.

### 4.2. Analysis of the Influence of Age on Patients with Respiratory Failure

The age of the patients with respiratory failure selected in this study is roughly between 58 and 75 years old. The differences were compared by multigroup analysis of variance. The total score of mechanical ventilation system efficiency evaluation was taken as the dependent variable, and the influence of the age of patients with respiratory failure was analyzed to study whether it has statistical significance. The data of patients with respiratory failure who participated in this study were compared, and the results are shown in Table 3.

It can be seen from Table 3 that there is a significant difference in the effectiveness evaluation of mechanical ventilation system among patients of different ages (*P* < 0.01), and there is a significant difference in the effectiveness of mechanical ventilation system among patients of different ages.

### 4.3. Analysis of Arterial Blood Gas in Patients with Respiratory Failure

Patients with respiratory failure have a high probability of relapse after the onset, so in the process of nursing, we need to pay attention to the mechanical ventilation oxygen therapy, which will have a beneficial impact on hemodynamics. Proper nursing has obvious curative effect on the symptoms of patients with respiratory failure. The arterial blood of the two groups of research objects was extracted before discharge, one month and six months after discharge, and the blood gas analysis indexes PH, pO_2_, and pCO_2_ were detected and recorded. The results are shown in Figure 1.

It can be seen from Figure 1 that the arterial blood gas of group A with comprehensive nursing is better than that of group B with general nursing. There was no doubt that the PH value of the two groups changed significantly 6 months after discharge. The pO_2_ value of group A was higher than that before discharge, while the pCO_2_ value of group B was unstable, and the pCO_2_ value was increased. The pO_2_ value of group A was 55.52 before discharge, and 62.36 six months after discharge. The pCO_2_ value of group A was 54.31 before discharge, and 50.61 six months after discharge. The pCO_2_ value of group B was 55.23 before discharge and 57.34 six months after discharge.

### 4.4. Analysis of Pulmonary Function Changes in Patients with Respiratory Failure

After the onset of respiratory failure patients, their lung function decreased significantly, and their activity ability was poor. In the case of comprehensive nursing, their lung function was better than that of ordinary nursing patients. In this paper, the lung function of two groups of patients was measured, and their forced vital capacity (FVC) and deep inspiratory capacity (IC) were taken as the analysis indexes respectively. The lung functions of patients before discharge, one month and six months after discharge, were tested, and the results are shown in Figure 2.

It can be seen from Figure 2 that the lung function of group A with comprehensive nursing is better than that of group B with general nursing. Group A was under comprehensive nursing, the data volume of FVC and IC increased after discharge, and their lung function recovered slowly. In group B, the data volume of FVC and IC decreased slowly, and their lung function began to decline.

### 4.5. Comparative Analysis of Treatment and Recovery

Respiratory failure patients gradually recover in the process of intensive care, but the recovery is not the same with different nursing methods. This study compared group A and B of patients with respiratory failure treatment recovery, from the patients with respiratory function recovery time, hospitalization time, and first second expiratory volume (FEV1), three aspects to compare the treatment effect of two groups of patients. The results are shown in Figure 3.

It can be seen from Figure 3 that the recovery time of respiratory function and hospitalization time of group A are shorter than those of group B, and the first second expiratory volume of group A is larger than that of group B. The average recovery time of respiratory function in group A was 5.13 days, while that in group B was 8.67 days, 23 days in group A, while 13.34 days in group B. The first second expiratory volume was 2.38 in group A and 1.94 in group B.

### 4.6. Analysis of Nursing Satisfaction of Patients with Respiratory Failure

Before the discharge of patients with respiratory failure, this study counted the satisfaction of patients with respiratory failure to the nursing staff and understood whether the nursing staff's actions in the nursing process satisfied the patients. The data results are shown in Table 4.

It can be seen from Figure 4 that in the nursing satisfaction results of patients with respiratory failure, the nursing satisfaction rate of group A is higher than that of group B. It can be seen that comprehensive nursing brings better body feeling to patients with respiratory failure.

## 5. Conclusions

Respiratory failure as a clinical respiratory disease needs more stringent care procedures, with its rapid onset, high risk, the number of times into intensive care, and the requirements of intensive care. The implementation of comprehensive nursing for patients can control the patient's condition and reduce the burden of patients with respiratory failure, which is widely favored by patients. The results of this study also show that the condition of patients with comprehensive nursing scheme is better than that of patients with general nursing, and comprehensive nursing has a good effect on patients with respiratory failure. Artificial intelligence is a branch of computer science. It attempts to understand the essence of intelligence and produce a new intelligent machine that can respond in a similar way to human intelligence. The research in this field includes robot, language recognition, image recognition, natural language processing, and expert system.

## Figures and Tables

**Figure 1:** Analysis of arterial blood gas in patients with respiratory failure.

**Figure 2:** Changes of pulmonary function in patients with respiratory failure.

**Figure 3:** Comparison of treatment and recovery.

**Figure 4:** Analysis of nursing satisfaction of patients with respiratory failure.

**Table 1:** Patient general information sheet.

	A group	B group	*P*
Gender (female: male)	8 : 17	12 : 13	*P* > 0.05
Age	67.1 ± 8.88	67.2 ± 7.73	*P* > 0.05
There is endotracheal intubation	1	1	*P* > 0.05
History of noninvasive ventilator	1	2	*P* > 0.05
History of family oxygen therapy	7	6	*P* > 0.05
pH	7.39 ± 0.05	7.41 ± 0.07	*P* > 0.05
PaCO_2_	43.1 ± 3.03	43.3 ± 4.14	*P* > 0.05
PaO_2_	95.41 ± 10.92	95.8 ± 11.45	*P* > 0.05
SpO_2_	94.5 ± 4.25	93.8 ± 4.37	*P* > 0.05

**Table 2:** Analysis of gender influence in patients with respiratory failure.

Gender	Number	Total efficiency
Male	30	13.16 ± 0.97
Female	20	13.92 ± 0.61
*P*		>0.05

**Table 3:** Analysis of the influence of age on patients with respiratory failure.

Age	Number	Total efficiency
55–60	13	13.24 ± 1.4
61–65	15	13.55 ± 1.32
66–70	14	13.2 ± 1.27
71–75	8	12.97 ± 1.48
*P*		<0.01

**Table 4:** Analysis of nursing satisfaction of patients with respiratory failure.

	Very satisfied	Quite satisfied	Dissatisfied	Total satisfaction
A group	46	3	1	49
B group	35	8	7	43

## Data Availability

The data underlying the results presented in the study are available within the manuscript.
